RETRACTED

# Construction of Digital Platform of Religious and Cultural Resources Using Deep Learning and Its Big Data Analysis

**DOI:** 10.1155/2022/4258577

**Published:** 2022-07-30

**Authors:** Qian Sun

**Affiliations:** School of Political Science and Public Administration, Shandong University, Qingdao 266237, China

## Abstract

This article analyzes the difficulties associated with the preservation and transmission of religious cultural resources and the difficulties encountered in the new development environment and background. It does so in light of the current state of religious, cultural resources. The protection, growth, and use of religious and cultural resources against the backdrop of the digital era are elaborated upon and critically analyzed in this article. Based on the foregoing discussion, this article conducts a thorough analysis of the development of a digital platform for religious and cultural resources and its big data analysis, and it also suggests an image feature extraction algorithm based on DL. This article develops a clustering CNN based on the network with PCA vector as convolution kernel, which clusters small images and computes principal component vectors according to categories, generating multiple groups of convolution kernels to extract more features so that the input image can select feature extractors adaptively. Simulation and comparative analysis are used in this article to confirm the algorithm's effectiveness. Compared to the conventional NN algorithm, simulation results indicate that this algorithm is more accurate, with a maximum accuracy of about 95.14 percent. It has some reference value for the research that will be done in relation to the creation of the next digital platform for religious and cultural resources.

## 1. Introduction

In today's society, religious resources are a rare and valuable wealth. An important task before us is to figure out how to develop and use them in a rational and efficient manner to support social development in the present [1]. To restore the glory of national culture, it is also necessary to unearth outstanding traditional religious cultural resources and to encourage their imaginative transformation and innovative development. Many people today still reject religion as superstition and ignorance and completely discount its cultural significance [2]. The issues that need to be taken into consideration at this point include how to use new media to promote and disseminate religious cultural resources, how to better integrate digital technology with religious cultural industries, how to speed up the development of nonreligious cultural industries, and how to encourage the protection, inheritance, and development of religious cultural resources. First and foremost, religious resources are a subset of resources for religious belief. People who have mastered religious ideas and concepts are eager to contribute to the cause, so they band together to found religious organizations and engage in a variety of religious activities [3]. People's lives move quickly in the new media era, so they are more willing to read content that presents information in a more logical and effective way. When compared to other types of information, visual senses, which are a relatively direct channel for receiving human information, can be used to convey information to readers [4]. Audience members can sense the allure of religious culture because the image is presented to them with a vivid image and a real voice. The “original ecology” of religious culture is embodied by the comprehensive application of image, sound, picture, and other elements and symbols that is presented in a unified way of time and space. It has obvious agility and authenticity when compared to traditional language communication and graphic picture communication.

RETRACTED

The public's spiritual and cultural needs are growing daily, and the standards for cultural experiences are also improving to previously unheard-of levels. Although there are still some gaps in its transformation and application in production and daily life, the excavation of religious cultural resources is currently primarily manifested in inheritance and protection, and the path of industrial transformation is primarily focused on religious tourism. It can't better meet the fervent spiritual and cultural needs of the populace because it ignores cultural connotation, lacks innovative ideas, and is in a primary state overall. The path of creative transformation of religious and cultural resources should therefore be broadened. The text image processing of traditional cultural images is just one aspect of the narrative communication of traditional cultural images; other aspects include the preservation and advancement of traditional cultural images and information technology. Therefore, interdisciplinary related work is essential to effectively communicating traditional culture. The digitization of religious culture must be upgraded from the initial low-level digitization of the most basic written materials and audio and video materials to the knowledge and big data of religious culture in order to provide massive data resources for the creation of cultural digital platforms. This upgrade is required in light of the development of big data, cloud computing, and Internet of Things technology [5]. The idea of DL (deep learning) [6, 7] was created during the artificial neural network [8, 9] research process. A multilayer perceptron called NN is made up of a lot of artificial neurons that are connected to one another. The value of corresponding technology for applications is increasing along with the ongoing development of DL and AI. Applications built on NN technology are now competitive in a number of industries. They are also increasingly used in the fields of semantic understanding and image recognition. DL is a collection of different NNs. These NNs are incredibly numerous and intricate, and the hierarchical structure is astounding. Unlike feature extraction in conventional machine learning, feature extraction based on deep learning (DL) can also extract the images' high-level semantic information in addition to their basic features. As a result, one of the hot areas in the current image field is the research of feature extraction based on DL [10]. The development of a digital platform for religious and cultural resources, as well as its big data analysis, is thoroughly examined in this article. Additionally, a proposed image feature extraction algorithm based on DL is put forth. The following are the innovations of this article:

1. Aiming at the limitation of traditional feature point extraction algorithm, this article proposes an image feature point extraction method based on NN based on DL technology to improve the feature point detection ability. At the same time, this article proposes a feature selection method based on semisupervised ladder network. This method solves the training problem of unlabeled data samples through the ladder loss function and improves the retrieval efficiency by combining the four-value hash retrieval algorithm.
2. In this article, feature extraction models based on directional gradient histogram, scale-invariant feature transformation, and CNN (Convolution neural network) are used to extract features from data, and the results are analyzed. The research shows that this network can extract multiple key region features of each image and use them for image retrieval, which effectively improves the efficiency and accuracy of image retrieval.

RETRACTED

## 2. Related Work

Wanyan and Dai proposed to reconstruct the intangible cultural heritage information by means of digital technology to adapt to the modern information environment under the condition of changing the original environment of the intangible cultural heritage and promote the informatization survival and development of the intangible cultural heritage [11]. Tsivolas pointed out that with the changes in the living conditions of cultural heritage and the rapid development of science and technology, many traditional protection methods are no longer suitable, and new protection methods are needed to replace them. Digital protection technology is one of the fastest developing and most concerned [12]. Wang et al. took traditional folk culture as the research object and the traditional cultural knowledge system as the research scope and explored the digital methods and means of traditional folk culture based on big data processing technology, so as to realize the visualization of folk data [13]. Pathak and Selvakumar analyzed the technical, semantic, and validity problems of intangible cultural heritage information dissemination in detail based on the needs for digital expression and diffusion of intangible cultural heritage information [14]. Li et al. summarized the relevant academic history and clues of the digitization of cultural resources in the era of big data from both domestic and international dimensions, clarifying that the digitization of cultural resources is the digital expression of the folk custom process through the collision and integration of culture and technology. Then they pointed out the next development path of the digitization of traditional cultural resources [15]. Deng and Xie reviewed and discussed the international and domestic research in the field of digital protection technology for tangible and intangible cultural heritage from the aspects of digital preservation and archiving of cultural heritage [16]. Hu and Xiao pointed out that the traditional color image edge feature extraction only utilizes middle-level and low-level information, and the edge feature extraction effect is not good. To this end, a multifeature color image edge feature extraction method that can utilize high-level information is proposed [17]. Beel et al. conducted an in-depth study of several classic CNNs, summarizing the way convolutional network models are developed. At the same time, an existing self-supervised learning feature point detection model is deeply explored, and an improved method for its shared convolutional layer is proposed [18]. In terms of the generation algorithm of convolution kernels, Pietrobruno first introduced the backpropagation algorithm in CNN and then introduced two kinds of autoencoder networks and deep belief networks that can be used for feature extraction and can be used to generate pretrained convolution kernels [19]. Yi et al. proposed two DL network structures for feature extraction in image retrieval: an image retrieval network based on clustered attention NN and an image hash retrieval network based on semisupervised ladder network [20]. The experimental results show that the image hash retrieval algorithm based on semisupervised ladder network has a certain improvement in accuracy and time efficiency, and the image retrieval algorithm based on clustering attention NN has a significant improvement in accuracy.

RETRACTED

This article elaborates and analyzes the preservation, advancement, and use of religious and cultural resources based on a thorough analysis of prior literature, and it also suggests a DL-based image feature extraction algorithm. This article suggests an image feature point extraction method based on NN based on DL technology to improve the feature point detection ability in order to address the shortcomings of conventional feature point extraction algorithms. According to the research, this network can extract several important region features from each image and use them to enhance image retrieval's accuracy and efficiency.

## 3. Methodology

### 3.1. Digitization of Religious Cultural Resources

As a theory of religious thought, religious culture has its own unique world outlook, outlook on life, and practice. Religion is not only a world outlook, outlook on life, and practice, but also its ideological theory is full of the wisdom of life. Relevant personnel should dig deep into the ideological concepts, humanistic spirit, and moral norms contained in excellent traditional culture, inherit and innovate according to the requirements of the times, and let the culture show its permanent charm and style of the times. They promote the creative transformation and innovative development of excellent religious culture and constantly create new cultural glory [21]. With the trend that digital technology is increasingly helping humanities research, it is becoming a new direction and a new topic for scholars to explore how to store and develop religious and cultural resources by digital means and build a database of humanities resources to assist academic research. At present, the research on religious culture has not received due attention, the organization is not perfect, the research strength of religious culture is weak, the research scope is not wide, and the research level is still relatively shallow. By visualizing traditional cultural texts and combining the use of new media platforms, people can now use the quickly evolving new media to further the spread of religious culture and encourage the growth of the social culture. The “Internet plus” era and big data present a good opportunity for the quick creation and dissemination of images. The advancement of new media has been encouraged by the times, and this advancement has altered the current media communication landscape. Images gradually demonstrate the benefits and ease of new media communication. Images can be used more effectively in a variety of fields where there is a need for information dissemination because they are more self-explanatory and can aid viewers in interpreting the narrative content of images across a time barrier. Image is a research method in and of itself, in addition to being a method of recording. New media introduces fresh viewpoints, materials, and ways of thinking.

RETRACTED

Religion is a type of cultural system as well as a type of belief. Religion has left a rich cultural legacy for humanity over thousands of years of history, which is represented by historical artefacts in physical form and intangible cultural heritage in nonphysical form. Religious heritage is on the verge of extinction and serves as a tangible expression of past knowledge, whether it be material or immaterial. We now have some better methods for tasks that the unified protection method cannot handle, thanks to the advancement of digital technology. Through digital technology, some extinct cultures can prolong their existence. Religion requires inheritors to realize the practice and inheritance of cultural heritage due to its singular immateriality. It is necessary to combine the actual situation of recorded inheritors and “nonlegacy” projects in order to create a shooting scheme that can accurately reflect the inheritors' practical ability and characteristics because all types of religious and cultural resources have their own characteristics and laws [22]. Religion is diverse and vibrant, with many different forms, and the cultural heritage materials of each region will vary slightly. When gathering and sorting materials, you can first put them into different categories based on the forming factors. For example, phonetic religious and cultural resources can be collected by electronic recording; the dynamic materials of songs and dances are collected by video collection and transmission of people's experiences. Then, it is classified according to factors such as humanistic characteristics, regional characteristics, ethical characteristics, and causal characteristics, so as to follow up the modeling of religious culture ontology. The digital application of material and intangible cultural heritage is shown in Figure 1.

Transforming religious and cultural resources into realistic material and spiritual productivity and developing various forms of religious and cultural industrial forms and projects are new bright spots in the development of cultural industry, an important manifestation of cultural prosperity and development, and an important engine to create a new growth point of the regional economy. As the religious cultural heritage itself is facing an endangered situation, it is an important strategy for the protection of religious cultural heritage to adopt advanced computer technology to combine its information sorting, monitoring, management, and decision-making, make a true, systematic and comprehensive record of precious, endangered, and historical religious cultural resources, and make virtual representation and establish permanent archives and databases. The distributed processing system is used to digitize, organize, and know large traditional cultural resources based on the integration platform of religious and cultural knowledge map, offering platform support and technical assistance for the realization of digital culture. With the rise of the digital age, visualization has emerged as a fresh method for many religious and cultural studies to preserve and promote traditional cultural heritage. The existing traditional religious cultural resources don't contain much-structured knowledge other than some simple written materials. It is challenging to directly apply religious cultural resources to the study of religious cultural maps because they are typically reflected in numerous WEB pages and self-media documents. Digital protection has many benefits over conventional methods. Traditional information storage media are expensive and have a limited amount of storage space. In addition to being inexpensive, digital archiving also has the advantage of storing more data than all previous eras combined. Digital technology is required if you want to fully preserve the knowledge of cultural heritage. Virtual images are a type of projection technology that creates an immersive experience for viewers by simulating real-world images and scenes on computers. It is a form of communication that primarily uses audio and video to express and convey ideas. The thorough integration of multimedia and multidimensional data and information allows for the omnidirectional and three-dimensional presentation of humanistic phenomena, conforms to the complexity characteristics of humanistic phenomena, and aids in stimulating researchers' ideas and facilitating multidimensional thinking and research on religious and cultural resources.

RETRACTED

### 3.2. Realization of Image Feature Extraction Algorithm Based on DL

It is one of the most important network models in CNN DL, an extremely effective network model, and plays an important role in image recognition and retrieval. CNN optimized the network structure, combined with local sensing, weight sharing, and pool down sampling to ensure the invariance of displacement. The convolution network has played an important role in the history of DL, and it is one of the first deep networks that can be effectively trained by backpropagation. The convolution kernel is a feature extractor in CNN, which extracts image features by sliding the convolution kernel on the image. The input interface of NN can be directly connected with the image, which reduces the complexity of feature extraction and data reconstruction in traditional image recognition algorithms and thus simplifies the operation process in terms of network input. NN can extract image features, including color, texture, shape, and topological structure of the image, etc. It has good robustness and work efficiency in identifying displacement, scaling, and other forms of distortion invariance. The image retrieval method based on DL makes use of a large amount of data in the image database, extracts image features through the NN model, and then saves them in the image database. When retrieving images, NN is used to extract the features of the images to be detected, and the similarity between the features of the images to be detected and those in the database is calculated. Finally, *N* similar images are output. The DL model and training process are shown in Figure 2.

The ability to detect feature points is enhanced in this article by the proposal of an image feature point extraction method based on NN. In NN, the image is primarily processed by convolution, which involves assigning a linear weight to each pixel. Not all issues in the real world are linear issues. We can intentionally add nonlinear factors to solve the issue that linear models are not universal, or we can convert nonlinear problems into linear problems in order to effectively resolve this situation. High-dimensional data can be reduced in dimension using the PCA (Principal Component Analysis) technique. The original data are projected into the new coordinate system after the new coordinate vector has been determined, with the goal of maximizing the variance of the projection data's first dimension in the new coordinate system. It is possible to omit the values in the dimension with the lower order, realizing dimension reduction, because as the dimension increases, the variance of the data in this dimension decreases in turn. The image to be retrieved is preprocessed, the image features are extracted, the feature vectors of the target image are compared to the feature vectors in the target image feature database by a superior similarity measurement algorithm, and finally, the retrieval results are sorted according to the similarity measurement results, and the retrieval results are obtained and output. To extract features, choose a picture from a dataset. To determine the pertinent parameters of feature transformation features with constant scale, it is necessary to have a general understanding of the dimensions of the obtained feature data. When the feature extraction scheme is put into practice, the parameters can be designed in accordance with the data structure and data type chosen in this paper. The quantity represents the optimal number of feature points that the algorithm, after ranking the detected feature points, has returned. The first step in the PCA network's training process is to PCA the training data. It should be noted that the original picture is not calculated in this case; instead, the small picture, whose dimensions match those of the convolution kernel, is first extracted from all of the training images. The convolution kernel of the first layer network will be the principal component vector of small picture data. The core layer in NN, the convolution layer, is responsible for extracting features from images. The feature map is produced by convolving the image with the convolution kernel in the convolution layer. An independent feature detector in an image is a convolution kernel. Each convolution layer's output feature graphs are represented by the number of convolution kernels in that layer. Calculate the mean value using the following formula for the initial feature sample:

(1) $$\begin{array}{c} \mu_{\lambda }=\frac{\sum_{i=1}^{m}x_{i}}{m}. \end{array}$$

We compute the feature sample variance based on the mean:

(2) $$\begin{array}{c} \sigma_{\lambda }^{2}=\frac{\sum_{i=1}^{m}{\left(x_{i}-\mu_{\lambda }\right)}^{2}}{m}. \end{array}$$

Normalization is done by the following:

(3) $$\begin{array}{c} \bar{x_{i}}=\frac{x_{i}-\mu_{\lambda }}{\sqrt{\sigma_{\lambda }^{2}+\varepsilon }}. \end{array}$$

In the formula, *λ* is used to describe the minimum batch value. Batch normalization needs to process all training data at the same time, which is almost impossible in practical applications, so only the data in the current iteration is processed. *ε* stands for a very small number and is used to avoid situations where the denominator is 0.

RETRACTED

Suppose the dataset has *I* samples, the sample dimension is *J*, it is represented as a data matrix *X*, and then *X* is the *I* × *J* dimension matrix, that is,

(4) $$\begin{array}{c} X=\left[\begin{array}{c} x_{1}^{T}\\ x_{2}^{T}\\ \ldots \\ x_{I}^{T} \end{array}\right]={\left[\begin{array}{cccc} x_{1,1}, & x_{1,2}, & \ldots , & x_{1,J}\\ x_{2,1}, & x_{2,2}, & \ldots , & x_{2,J}\\ \ldots & \ldots & \ldots & \ldots \\ x_{I,1}, & x_{I,1}, & \ldots & x_{I,J} \end{array}\right]}_{I\times J}. \end{array}$$

Here, $x_{i}=\left[\begin{array}{c} x_{i,1}\\ x_{i,2}\\ \ldots \\ x_{i,J} \end{array}\right]$ represents the *i*th sample. Since we want the data to fluctuate the most on the axis represented by the principal components, the sum of squares projected on *u* for all samples is the largest, as shown in the following formula:

(5) $$\begin{array}{c} u^{*}=\arg\max\frac{1}{I}{\sum_{i=1}^{I}\left(x_{i}^{T}u\right)}^{2}=\arg\max u^{T}\left(\frac{1}{I}\sum_{i=1}^{I}x_{i}x_{i}^{T}\right)u. \end{array}$$

If ∑=1/*I*∑_*i*=1_^*I*^*x*_*i*_*x*_*i*_^*T*^, then Σ is the covariance matrix of *X*, so the above formula becomes as follows:

(6) $$\begin{array}{c} u^{*}=\arg\max u^{T}\Sigma u. \end{array}$$

The parameter initialization operation can make the network structure train hundreds of layers without overfitting:

(7) $$\begin{array}{c} I*X=X,\\ I\left(i,j,l_{1},l_{2},l_{3},\ldots ,l_{L}\right)=\left\{\begin{array}{c} 1,\;\text{if }i=j,\\ 0,\;\text{otherwise.} \end{array}\right. \end{array}$$

Here, *I* represents the identity matrix of the same dimension as the input feature map, *X* represents the input feature map, and *i* and *j* represent the length and width of the input feature map, respectively. Obviously, when *I* is the unit matrix, the input feature map and the output feature map are the same, so the unit matrix *I* can be used as the convolution kernel to convolve the feature map to ensure that the original feature map is transmitted unchanged. The network convolution is designed as follows:

(8) $$\begin{array}{c} W\_1=\text{diag}\left(a\right)I+\text{diag}\left(b\right)W_{\text{norm}},\\ y=W\_1*X, \end{array}$$

where *X* is the input feature map and *W*_1 is the convolution weight.

When performing feature fitting, for the class sample dataset, feature fusion is mainly to aggregate the same samples and separate different samples. In order to avoid overfitting, a regular term is introduced into the feature fusion algorithm. Then, the edge feature fusion algorithm is given:

(9) $$\begin{array}{c} \underset{v}{\max}\frac{v^{T}Z_{b}v}{v^{T}Z_{t}v+\gamma_{1}v^{T}v+\gamma_{2}G\left(v\right)}. \end{array}$$

Here, *Z*_*b*_ and *Z*_*t*_ are used to describe the interclass divergence and overall divergence of the sample set in turn, and the formulas are as follows:

(10) $$\begin{array}{c} Z_{b}=\frac{\sum_{i=1}^{c}\left(m_{i}-m\right){\left(m_{i}-m\right)}^{T}}{n},\\ Z_{t}=\frac{\sum_{i=1}^{c}\left(x_{i}-m\right){\left(x_{i}-m\right)}^{T}}{n}. \end{array}$$

Here, *m*_*i*_ and *m* are used to describe the mean value of the samples of class *i* and all samples in turn; *v*^*T*^*v* is used to describe the regular term; *G*(*v*) is used to describe the prior knowledge; *γ*_1_ and *γ*_2_ are both constants higher than 0.

The goal of the similarity measure is to determine how similar the feature vectors of the image to be retrieved and the image in the database are. Choosing the right measurement technique is particularly crucial. Typically, the similarity increases with the proximity of the two vectors' directions and sizes. Since the small pictures in every position of every image are extracted in this study, it can be said that the small pictures hold all the image data, including texture, corners, and contours. If the images can be categorized using this data, PCA can be carried out by class. In this study, the classification number is changed to the appropriate number, the final full connection layer is eliminated, feature extraction is carried out, all candidate frames of the image are extracted, selective search is carried out, each region's size is changed to fit the network's input, a forward operation is carried out, the output of the fifth pool layer is made, and the features extracted from the candidate frames are stored. It's important to determine how similar the image features that need to be retrieved are to the image features stored in the database when performing image retrieval. The efficiency of the retrieval time is impacted by a large number of database images and the large image feature dimension in the actual retrieval process. The time efficiency of image retrieval can be increased by using hash retrieval, which maps high-dimensional features into low-dimensional hash codes. In this study, high-pass filtering is used to extract high-frequency images from the image, after which small images in the high-frequency image domain are extracted and clustered. This is because high-frequency filters are used in image restoration to develop a better dictionary for expressing local features and can improve meaningful features in low-level image processing. The output point actually matches the probability of an input point for feature point detection. A pair of encoders and decoders are present in the typical detection network. The image's dimension can be decreased, and the encoder can first extract the image's feature data. The low-dimensional output tensor is restored to the input's dimension by the decoder. Enough neurons are used in the entire connection layer to integrate the features that different neurons in the previous convolution layer extracted to form a feature vector. The primary purposes of CNN are the detection of displacement, scale changes, and other graphic distortions. When using CNN, the feature detection layer does not use manual feature extraction but instead directly learns from the training data.

RETRACTED

## 4. Result Analysis and Discussion

The training model for CNN must be trained beforehand. Training rarely begins at the top layer in general practical work training. Instead, the parameters of the layers in front of the model are fixed after the model has been trained beforehand on a large dataset. The final outcome will typically be excellent because only the final layers are changed when dealing with the current problems, and the data of the current problems are fine-tuned. This model's training procedure can be broken down into three steps: first, create a basic synthetic dataset for training the detector of interest points. The interest points are clearly and unambiguously placed on the synthetic dataset, which is composed of straightforward geometric shapes. The image is then detected using the basic detector, the unlabeled image is automatically marked using the homography transformation, and the labeled dataset is created. The full convolution network is then retrained using the tag data set created in the previous step. Only three cases with the best model convergence in the training results are provided as a result of numerous experiments.  Figure 3 displays the outcomes of the network training.

Compared with ordinary color images, the image information of gray-scale images is relatively much less, and it also takes up less storage space in the computer. Therefore, in image processing, color images can be converted into gray-scale images first so that the calculation amount can be relatively reduced and more computing power can be applied to other links. In this article, after obtaining the set of small images, we use the following clustering rules: set the variance threshold and divide all small images whose variance is less than the threshold into class 0, which are smooth images. This operation keeps the meaningful feature pictures, which is beneficial to the subsequent clustering. The experimental parameter settings in this chapter are shown in Table 1.

The comparison algorithm code in the experiment mainly comes from the open source DNNH. Data cleaning tools include two cleaning schemes: intraclass data cleaning and interclass data cleaning. Intraclass data cleaning is to cluster the same class of data by using a clustering algorithm. If the number of clusters in the clustering result exceeds 1, it means that there is noise data in this class of data that needs to be cleaned. Feature extraction of the image target object by scale-invariant feature transformation is conducted. In this article, OpenCV software is used to realize the method of classifying image objects by sifting, which comes from the realization of classic word bags. Before the implementation, you must first set the input format and the storage location of the input training data folder.

RETRACTED

Accuracy and recall reflect two aspects of classifier performance. In this article, the image feature extraction method based on directional gradient histogram, the image feature extraction method based on scale-invariant feature transformation, and this method are compared and tested. The accuracy results of different methods are shown in Figure 4. The recall results of different methods are shown in Figure 5.

It can be seen that the accuracy and recall of this method are both at a high level. In order to evaluate a classifier more comprehensively, this article chooses to introduce F1-Score as a comprehensive index. The F1-Score test results of different algorithms are shown in Figure 6.

When the data training samples are few, the recognition error rate of this network is lower than that of others. This is because its model is simple, with only three layers of networks, and its parameters are far smaller than those of other networks, so it is not easy to fall into overfitting. In essence, the convolution kernel of this network is pretrained, so it has good recognition ability. Using different methods and different data sets for testing, the average accuracy of feature extraction is shown in Table 2.

After observing the three feature extraction methods, it is found that the accuracy of the feature extraction method based on DL is better than that of the traditional feature extraction method. This is because the traditional feature extraction method is a unique algorithm designed by previous people for a specific environment, while the feature extraction method based on DL can obtain an extraction scheme that is more suitable for the environment through continuous self-learning, thus obtaining a favorable situation. The test running time on the model dataset is shown in Figure 7.

In terms of running time, the running time of PCANet is slightly higher than that of the network in this article, but since the network in this article and PCANet do not need to use a backpropagation algorithm to learn parameters, their time consumption is lower than that of other comparative experimental models. In order to verify the performance of the algorithm, this section makes a comparative analysis of the simulation. Simulation results show that the accuracy of this algorithm can reach about 95.14%. The results show that the accuracy of the image feature extraction method based on DL is higher than that of the image feature extraction method based on machine learning under normal conditions, both after image gray level normalization and under the condition of uncertain angle.

## 5. Conclusions

Religion is a unique cultural phenomenon that has shaped the evolution of human society and is a significant component of traditional human culture. It has an effect on society's economic and cultural life in addition to the spiritual lives of religious believers. In today's society, religious resources are a rare and valuable wealth. An important task before us is to figure out how to develop and use them in a rational and efficient manner to support contemporary social development. The digitization of religious culture must be upgraded from the initial low-level digitization of the most basic written materials and audio and video materials to the knowledge and big data of religious culture in order to provide massive data resources for the creation of cultural digital platforms. This upgrade is required in light of the development of big data, cloud computing, and Internet of Things technology. This article suggests a DL-based image feature extraction algorithm based on a thorough analysis of prior literature. This article suggests an image feature point extraction method based on NN based on DL technology to improve the feature point detection ability in order to address the shortcomings of conventional feature point extraction algorithms. This article uses feature extraction models based on directional gradient histogram, scale-invariant feature transformation, and CNN to extract features from data and analyses the outcomes to verify the algorithm's performance. The experiment validates the efficacy of this method, and the simulation results show that the accuracy of this algorithm can reach about 95.14 percent. The research results show that the accuracy of the image feature extraction method based on DL is higher than that of the image feature extraction method based on machine learning under normal conditions, after image gray level normalization, and under the condition of uncertain angle. It has certain reference significance for the subsequent research on the construction of digital platforms of religious and cultural resources.

RETRACTED

## Figures and Tables

**Figure 1:** Digital application of material and intangible cultural heritage.

**Figure 2:** DL model and training process.

**Figure 3:** Network training results.

**Figure 4:** Accuracy test results of different algorithms.

**Figure 5:** Test results of recall rate of different algorithms.

**Figure 6:** F1-Score test results of different algorithms.

**Figure 7:** Comparison of the model running time.

**Table 1:** Experimental parameter setting.

Project name	Specific parameters
Processor	Intel Core i7
Internal storage	16G
Operating system	Ubuntu
Development language	Python, C++
DL framework	MXNET
Learning rate	0.002
Weight attenuation	0.0005
Momentum value	0.9

**Table 2:** Average precision table of feature extraction.

Model	Dataset A	Dataset B	Dataset C	Dataset D
This article's network	0.841	0.801	0.847	0.871
PCANet	0.756	0.787	0.803	0.797
Scat-NET	0.692	0.669	0.691	0.695
GoogLeNet	0.567	0.594	0.621	0.689
Clustering attention net	0.789	0.791	0.754	0.799
DSH	0.691	0.687	0.679	0.691

## Data Availability

The data used to support the findings of this study are available from the author upon request.
